The article "Spare Parts Stocking Decision Strategy and Service Logistics Cost Optimization of Two-Echelon Service Logistics System considering Multifailure Mode" was retracted in 2023. Reasons: unreliable results or conclusions; concerns about the data; concerns about the peer review; concerns about the citations.

# Spare Parts Stocking Decision Strategy and Service Logistics Cost Optimization of Two-Echelon Service Logistics System considering Multifailure Mode

**DOI:** 10.1155/2022/7607985

**Published:** 2022-03-08

**Authors:** Ruiqi Wang, Guangyu Chen

**Affiliations:** School of Management and Economics, University of Electronic Science and Technology of China (UESTC), Chengdu, China

## Abstract

For the repair level and spare parts stocking decision problems, generally METRIC type methods and level of repair analysis (LORA) are used separately. In practical engineering, the repair level of large-scale systems is usually judged according to the failure modes. The method of judging the repair level by the maintenance success rate is no longer applicable. In the case of multiple failure modes of a large-scale system, considering the requirements of system availability, we build a spare parts stocking decision and service logistics cost optimization model of a two-echelon service logistics system. Aiming at the spare parts stocking allocation problem caused by multiple failure modes, we improve the iterative greedy heuristic algorithm to find the global optimal stocking allocation strategies. Finally, through the analysis of typical examples, the correctness and effectiveness of the model and algorithm are verified. The impact of multifailure mode spare parts stocking allocation strategies on availability and service logistics cost is analyzed. The research results are helpful to simplify the support engineering design process of system engineers and have certain theoretical and application value.

## 1. Introduction

Large-scale system can be decoupled or decomposed into multiple interrelated subsystems or modules. Each subsystem contains a variety of components, which are controlled by the same constraints or objectives to complete specific tasks. Therefore, any component's failure will cause system failure [1, 2]. The large number of components means that a reasonable service logistics strategy should be developed to meet the availability of spare parts and the economy of the service logistics system [3].

In terms of economy, due to the complex operational environment of large-scale system, the establishment of maintenance center for unified resource allocation and repair failure units could save a lot of costs compared to on-site maintenance [4]. In terms of availability, on-site maintenance would save the transportation waiting time of failed units and improve system availability [5]. Therefore, the aim of service logistics strategy is to balance the relationship between maintenance level, spare parts stocking allocation, and service logistics cost under the constraint of system availability.

The article "Spare Parts Stocking Decision Strategy and Service Logistics Cost Optimization of Two-Echelon Service Logistics System considering Multifailure Mode" was retracted in 2023. Reasons: unreliable results or conclusions; concerns about the data; concerns about the peer review; concerns about the citations.

The METRIC model is the most commonly used in service logistics strategy. The original METRIC model used “echelon” to represent the levels of different types of warehouses [6]. Slay [7] developed the VAR-METRIC model, which assumes that the average number of components in repair is equal to the variance of the negative binomial distribution. Graves [8] explored the same distribution, elaborating both an approximate and an exact method for the multiechelon single-indenture case. On this basis, literature [9] provides an accurate method to evaluate multiechelon service logistics systems. Therefore, the VAR-METRIC model is the most common method used by scholars to solve spare parts stocking allocation problems.

The level of repair analysis (LORA) is an input decision parameter of the VAR-METRIC model to solve the spare parts stocking allocation, and it is used to determine the location of spare parts for repair [10]. Falkner [11] was the first scholar to mention joint optimization of spare parts stocking decision and repair in his paper. Performing the LORA first and then the spare parts stocking decision analysis, the sequential approach, may lead to a solution that is not optimal. Basten [12] proposed an integrated algorithm to find optimal solutions for two-echelon problems. He uses efficient points on the curve of costs versus expected number of backorders to represent the optimal solution. On this basis, he proposed an iterative algorithm to solve the joint problem of LORA and spare parts stocking decision in 2015. The basic idea is to solve the LORA decision first, then use the VARI-METRIC model to solve the spare parts stocking decision problem, and last use the results of VARI-METRIC to add an estimate of the holding costs to the LORA inputs and start a second iteration [10]. However, all the above studies assume that component failure is a single failure mode.

Large-scale systems have a large number of components, leading to a large number of complex failure mechanisms. That is, different failure modes have different degrees of influence on the system [13]. To define or distinguish these failure modes, many scholars will choose failure mode analysis according to failure mechanism, failure impact, failure rate, or other parameters [14]. Failure mode analysis is an important work item of system availability analysis, and it is the basis for maintainability analysis, safety analysis, testability analysis, and supportability analysis [15]. Therefore, before formulating LRU maintenance level and spare parts stocking decision strategies, failure modes analysis of key component should be done first.

The introduction of multiple failure modes would change the joint optimization model of METRIC and LORA. Different echelon warehouses need different types of spare parts. Therefore, a new two-echelon service logistics cost optimization model for large-scale system is built in this paper. We improve an iterative greedy heuristic algorithm based on literature [10]. Finally, the correctness and effectiveness of the model and algorithm are verified by a practical engineering case. The key influencing factors of spare parts stocking allocation decisions and system availability are revealed. This research has certain theoretical and application value in the optimization of service logistics strategy.

The article "Spare Parts Stocking Decision Strategy and Service Logistics Cost Optimization of Two-Echelon Service Logistics System considering Multifailure Mode" was retracted in 2023. Reasons: unreliable results or conclusions; concerns about the data; concerns about the peer review; concerns about the citations.

## 2. Model Description

This section describes the characteristics of two-level support system for a large-scale operation system. According to the current research, we consider the influence of multiple failure modes on system operation results and the impact on maintenance strategy of support system. It provides a theoretical basis for the construction of the spare parts stocking decisions optimization model.

### 2.1. System Description

According to the hierarchical structure of Figure 1, this paper proposes a large-scale operation system with multiple failure modes. The system contains *k* identical individual subsystems, and each subsystem consists of *i* (*i* = 1, 2, 3,…) series components. LRU_*i*_ is the key component of the subsystem. In case of failure, it can be repaired at the maintenance site of the support system.

The structure of large-scale system is complex, and LRU often has a variety of failure modes FMi, *n* (*n* = 1, 2, 3,…) [16–18].

The key components of subsystems are various, including electronic, mechanical, and optical components. A single failure mode cannot meet the requirements of system availability analysis. At present, scholars generally use three classification methods: the impact of failure on components, the impact of failure on maintenance strategies, and the impact of failure on operating system. The first type divides the failure into degraded function failure, nonfunction failure, partial function failure, intermittent function failure, and unexpected function failure [19, 20]. The second type divides the failure into maintainable failure and nonmaintainable failure [21]. The third type divides failures into hard failure and soft failure [22–24].

Considering that our optimization model is a service logistics model, we pay more attention to the impact of spare parts stocking decision strategies on system operation results. Therefore, the third type is selected as the classification method in this paper. Soft failure usually causes system production reduction or inferior performance, while the system keeps functioning; hard failure can cause system failure, for example, the service logistics model of an offshore wind farm in literature [5]. According to the difficulty of maintenance caused by the marine environment and the impact of turbine failure on the system, hard failure and soft failure classification methods are used to formulate maintenance strategies for different failure modes.

The article "Spare Parts Stocking Decision Strategy and Service Logistics Cost Optimization of Two-Echelon Service Logistics System considering Multifailure Mode" was retracted in 2023. Reasons: unreliable results or conclusions; concerns about the data; concerns about the peer review; concerns about the citations.

Specifically, we ascribe the sudden failure modes such as circuit break, short circuit, and impact to hard failure, which will lead to the instantaneous loss of system function. We ascribe wear, aging, fatigue, and other degradation failure modes to soft failure, which reduces the key performance of the system. According to the above analysis, the basic assumptions of large-scale operation system in this study are as follows:

1. LRU_*i*_ (*i* = 1, 2, 3,…) are independent of each other, and the demand for spare parts follows the Poisson distribution.
2. System failure would be caused by one LRU at most. Multiple failures that occur at the same time are not considered.
3. When there is a shortage of spare parts in a failure maintenance site, the system stops, and the system availability decreases.
4. The importance of all LRUs is the same, and the priority is not considered for maintenance.
5. Failure diagnosis time and spare parts replacement time are ignored.
6. Each LRU has multiple failure modes FMi, *n* (*n* = 1, 2, 3,…). The failure modes are mutually exclusive; that is, the simultaneous occurrence of multiple failure modes is not considered.
7. Failure modes are divided into hard failure and soft failure.

### 2.2. Two-Echelon Service Logistics System Description

When the operating system fails, the corresponding failed spare parts shall be replaced immediately, and the removed failed spare parts shall be sent to the maintenance site for repair [17]. In the level of repair analysis (LORA), the expensive resource cost usually leads to the repair work upstream of the maintenance network, while the expensive transportation cost leads to the downstream repair work close to the installation Base. Therefore, spare parts with cheap resources should generally be repaired locally, while spare parts requiring expensive resources should be repaired intensively [16].

Considering that the hard failure is mainly caused by overload, instantaneous impact, and electronic failure, it is assumed that the “Base” site of the service logistics system can completely repair this failure mode. However, the soft failure needs to be reprocessed and assembled. In such cases, maintenance activities are expensive to deploy to the complex operating environment on the Base site. Therefore, we assume that the soft failed spare parts are sent to a higher-grade maintenance site “Depot.” In this study, the purpose of considering multiple failure modes is to solve the problem of choosing the maintenance position of multiple spare parts types, which can make up for the spare parts allocation problem that LORA can only solve a single failure mode. Using failure mode characteristics to determine the maintenance level is more suitable for practical engineering.

The article "Spare Parts Stocking Decision Strategy and Service Logistics Cost Optimization of Two-Echelon Service Logistics System considering Multifailure Mode" was retracted in 2023. Reasons: unreliable results or conclusions; concerns about the data; concerns about the peer review; concerns about the citations.

The maintenance activities at different maintenance sites are different. We consider a two-echelon service logistics system. This system's availability depends on the availability provided by any single maintenance site [17], and its structure is shown in Figure 2.

At each maintenance site of the service logistics system, maintenance resources such as maintenance tools, maintenance personnel, and support equipment are configured to enable it to deal with different failure modes. The Base is usually set at the site of the operating system. In case of failure, if the spare part is in stocking in the Base, the spare part shall be extracted and replaced immediately to restore system availability. If the spare parts are out of stocking, an order will be issued to the Depot, and an (*s* − 1, *s*) replenishment strategy will be formulated [12, 17].

The maintenance of failed spare parts requires inspection to determine the failure mode and relevant maintenance activities: LRU with hard failure is repaired in Base, and LRU with soft failure is repaired in Depot. The Depot can be regarded as a warehouse with unlimited capacity. However, due to cost control, we still need to optimize the amount of LRUs stored in maintenance sites. When the failed spare part is repaired in the Depot, it will be sent to the source Base again [16].

According to the above analysis, the basic assumptions of the two-echelon service logistics system are as follows:

1. The maintenance site has the maintenance ability to deal with the corresponding failure mode; that is, discard decision is not considered
2. The hard failure shall be repaired in Base, and the soft failure can only be repaired in Depot
3. Base and Depot deal with different failures, their resource allocation and maintenance difficulties are different, and the repair time of failures is independent
4. The maintenance strategy selects perfect maintenance; that is, LRU is repaired as good as new
5. There are no lateral transshipments between locations at the same echelon level or emergency shipments from locations at a higher echelon level
6. Maintenance resources are nonconsumables and can be reused

The purpose of failure mode classification is to distinguish the types of spare parts. Under different failure modes, LRU needs different types of spare parts, different maintenance difficulties, and different maintenance positions. The optimization model in this study is also applicable to other failure mode classification methods. As long as the failure mode characteristics can be determined, the maintenance level problem can be solved according to the maintenance requirements of spare parts.

The article "Spare Parts Stocking Decision Strategy and Service Logistics Cost Optimization of Two-Echelon Service Logistics System considering Multifailure Mode" was retracted in 2023. Reasons: unreliable results or conclusions; concerns about the data; concerns about the peer review; concerns about the citations.

## 3. Two-Echelon Service Logistics Cost Optimal Modelling

The purpose of constructing this optimization model is to find the spare parts stocking allocation strategy that makes the service logistics cost optimal under the condition of meeting the requirements of system availability. We improve the LORA and METRIC joint model and design a new iterative algorithm. The model variables are shown in Table 1.

### 3.1. Mathematical Model of Spare Parts Stocking Decision

Generally, a variable is defined in the METRIC model to represent the maintenance capability of the maintenance site, representing the probability of successful repair by LRU_*i*_ at *j*. This method is applicable to the case of single failure mode. In the case of multiple failure modes, the maintenance level should be determined in advance so that each maintenance point has sufficient capacity to deal with the current failure. This idea can not only clarify the resource allocation of different maintenance sites but also improve the efficiency of system availability management.

In this paper, the availability of the service logistics system is selected as the index to measure the effectiveness of the spare parts stocking decision [25]. The spare parts stocking holding cost optimization model of the two-echelon service logistics system is as follows:

(1) $$\begin{array}{c} \left\{\begin{array}{cc} \min, & \sum \sum fc_{i,j}\cdot s_{i,j},\\ s.t., & A\left(s_{i,j}\right)\geq A_{\text{min}}. \end{array}\right. \end{array}$$

Equation (1) indicates that the optimal spare parts stocking holding cost should meet the availability requirements *A*_min_.

When there are no LRU spare parts to be replaced in the warehouse of the maintenance site, the LRU will enter the shortage state, which will lead to the shutdown of the operating system and the decline of system availability. The relationship between availability and shortage of maintenance sties is as follows [26]:

(2) $$\begin{array}{c} A\left(s_{i,j}\right)={\left(1-\frac{\text{EBO}\left(s_{i,j}\right)}{M_{i,j}}\right)}^{M_{i,j}}, \end{array}$$

where *M*_*i*,*j*_ is the assembly quantity of LRU_*i*_ at *j*.

Since the failure of any LRU will cause system shutdown, it can be considered that the LRUs are in a series structure. The availability of the service logistics system  *A*_sys_ is the product of the availability of all maintenance sites:

(3) $$\begin{array}{c} A_{\text{sys}}=\overset{J}{\underset{j=1}{\prod }}\overset{I}{\underset{i=1}{\prod }}A\left(s_{i,j}\right)\\ =\overset{J}{\underset{j=1}{\prod }}\overset{I}{\underset{i=1}{\prod }}{\left(1-\frac{\text{EBO}\left(s_{i,j}\right)}{M_{i,j}}\right)}^{M_{i,j}}. \end{array}$$

Take logarithms on the left and right sides of (3) to obtain

(4) $$\begin{array}{c} \text{ln}\;A_{\text{sys}}=M_{i,j}\cdot \text{ln }1-\frac{\text{EBO}\left(s_{i,j}\right)}{M_{i,j}}\approx M_{i,j}\cdot -\frac{\text{EBO}\left(s_{i,j}\right)}{M_{i,j}}\\ =-\text{EBO}\left(s_{i,j}\right). \end{array}$$

Equation (4) can be simplified by using the equivalent infinitesimal principle. Because of *A*_sys_ ∈ [0,1] and EBO(*s*_*i*,*j*_) ≥ 0, finding the maximum value of system availability is equivalent to finding the minimum value of stocking shortage. Therefore, the solution of availability is transformed into the solution of stocking shortage and finally into the solution of the spare parts stocking decision of the service system [27].

The article "Spare Parts Stocking Decision Strategy and Service Logistics Cost Optimization of Two-Echelon Service Logistics System considering Multifailure Mode" was retracted in 2023. Reasons: unreliable results or conclusions; concerns about the data; concerns about the peer review; concerns about the citations.

EBO represents the LRUs' expected shortage when the service system stocking level is *s*_*i*,*j*_. EBO can be expressed as

(5) $$\begin{array}{c} \text{EBO}\left(s_{i,j}\right)=\sum_{\mathrm{x=}s_{\mathrm{i,j}}\mathrm{+1}}^{\infty }\left(x-s_{i,j}\right)p\left(x|N_{i,j}\right), \end{array}$$

where *N*_*i*,*j*_  is the intermediate variable of the optimization model. It represents the average number of LRUs in maintenance status. After maintenance activities, it can be provided to the system again as new spare parts for storage. According to the Palm theorem, when the LRU demand obeys the Poisson process with mean value *λ* and the mean repair time is *T*, the steady-state probability distribution of *N* obeys the Poisson distribution with the mean value *λT* [26]. That means

(6) $$\begin{array}{c} N=\lambda \cdot T. \end{array}$$

Set the number of LRU_*i*_ failures in a single cycle to *λ*_*i*_. After inspection, the number of hard failures is set to *λ*_*i*h_, and the number of soft failures is set to *λ*_*is*_. Their relationship can be expressed as follows:

(7) $$\begin{array}{c} \lambda_{i}=\lambda_{ih}+\lambda_{is}. \end{array}$$

In the case of multiple failure modes, the expected shortage of LRU_*i*_ should also be divided into Depot expected shortage EBO(*s*_*i*,0_) and Base expected shortage EBO(*s*_*i*,*j*_).

Since the failed spare parts in soft failure mode are repaired in Depot, the number of parts under repair in Depot is

(8) $$\begin{array}{c} N_{i,0}=\lambda_{is}\cdot T_{i,0}. \end{array}$$

Bring (8) into (5), and LRU_*i*_ expected shortage at the Depot is

(9) $$\begin{array}{c} \text{EBO}\left(s_{i,0}\right)=\sum_{\mathrm{x=}s_{i\mathrm{,0}}\mathrm{+1}}^{\infty }\left(x-s_{i,0}\right)p\left(x|\lambda_{is}\times T_{i,0}\right), \end{array}$$

where EBO(*s*_*i*,0_) is a stocking-related variable. When the operating system fails, a replenishment request is sent to the Base for the first time. If the Base is short of spare parts, a request would be sent to the Depot. Due to the ordering and transportation time *O*_*i*,*j*_, the number of spare parts under repair of Base *j* should consider transportation spare parts:

(10) $$\begin{array}{c} N_{i,j}=N_{i,j}^{1}+N_{i,j}^{2}. \end{array}$$

The number of parts under repair *N*_*i*,*j*_^1^ in Base is

(11) $$\begin{array}{c} N_{i,j}^{1}=\lambda_{ih,j}\cdot T_{i,j}. \end{array}$$

The number of parts under transportation *N*_*i*,*j*_^2^ should consider two situations:

(1) When Depot has spare parts stocking, the number of spare parts under repair is the number sent to Depot:
  (12) $$\begin{array}{c} N_{i,j}^{2^{\prime }}=\lambda_{is,j}\cdot O_{i,j}. \end{array}$$
(2) When the Depot is short of spare parts, the spare parts should be sent back to Base after being repaired at Depot. The average number of spare parts waiting for maintenance is equal to the expected shortage:
  (13) $$\begin{array}{c} N_{i,j}^{2\prime \prime }=\lambda_{is,j}\cdot f_{i,j}\cdot \frac{\text{EBO}\left(s_{i,0}|\lambda_{is}T_{i,0}\right)}{\lambda_{is}}, \end{array}$$
where  *f*_*i*,*j*_=*λ*_*is*,*j*_/*λ*_*is*_, which indicates the proportion of LRU_*i*_ sent by Base *j*. Based on the above analysis, the number of spare parts under repair in a single cycle can be expressed as
  (14) $$\begin{array}{c} N_{i,j}=N_{i,j}^{1}+N_{i,j}^{2\prime }+N_{i,j}^{2\prime \prime }\\ =\lambda_{ih,j}\cdot T_{i,j}+\lambda_{is,j}\left[O_{i,j}+\cdot f_{i,j}\cdot \frac{\text{EBO}\left(s_{i,0}|\lambda_{is}T_{i,0}\right)}{\lambda_{is}}\right]. \end{array}$$

Therefore, the expected shortage of Base is a variable related to stocking level and expected shortage of Depot:

(15) $$\begin{array}{c} \text{EBO}\left(s_{i,j}\right)=\sum_{\mathrm{x=}s_{\mathrm{i,j}}\mathrm{+1}}^{\infty }\left(x-s_{i,j}\right)p\left(x|N_{i,j}\right). \end{array}$$

The article "Spare Parts Stocking Decision Strategy and Service Logistics Cost Optimization of Two-Echelon Service Logistics System considering Multifailure Mode" was retracted in 2023. Reasons: unreliable results or conclusions; concerns about the data; concerns about the peer review; concerns about the citations.

### 3.2. Mathematical Model of Service Logistics Cost

The service logistics cost includes the spare parts stocking holding cost as well as maintenance cost and resource allocation cost. In general, maintenance cost and resource allocation cost are often defined in the LORA decision optimization model. If multiple failure modes are considered in service decisions, we find that the steps of iterating LORA model input variables can be simplified.

Maintenance service decisions usually include two kinds of decisions: on-site repair or move to repair. The decision cost can be expressed as *vc*_*i*,*j*,*d*_, *d* ∈ {repaire, move}. The resource allocation cost can be expressed as *rc*_*r*,*j*_ (*j*=1,  2,  3,…).

In the case of the single failure model, maintenance service decisions and resource allocation decisions are selected by the method of repeatedly iterating the possibility of all maintenance sites. In the case of multiple failure modes, we believe that different levels of maintenance site service different failure modes and configure different resources. Therefore, the LORA decision model can be simplified as

(16) $$\begin{array}{c} \text{min }\left[\sum \sum \lambda_{ih,j}\cdot vc_{i,j\text{,repair}}+\sum \sum \lambda_{is,j}\cdot \left(vc_{i,j,\text{move}}+vc_{i,0\text{,repair}}\right)+\sum \sum rc_{r,j}\right]. \end{array}$$

### 3.3. Mathematical Model of Spare Parts Stocking Decision Strategy and Service Logistics Cost

Combining (1) and (16), we can obtain the spare parts stocking decision strategy and service logistics cost optimization model:

(17) $$\begin{array}{c} s.t.\left\{\begin{array}{cc} \min & \left[\sum \sum fc_{i,j}\cdot s_{i,j}+\sum \sum \lambda_{ih,j}*vc_{i,j,\text{repair}}+\sum \sum \lambda_{is,j}*\left(vc_{i,j,\text{move}}+vc_{i,0,\text{repair}}\right)+\sum \sum rc_{r,j}\right],\\ s.t & \begin{array}{c} A\left(s_{i,j}\right)\geq A_{\text{min}}\;\left(i=1,2,3,\ldots ;\;j=0,\;1,\;2,\;3,\ldots \right),\\ \lambda_{ih}+\lambda_{is}=\lambda_{i}\;\left(i=1,2,3,\ldots \right). \end{array} \end{array}\right. \end{array}$$

Literature [12] designed an algorithm of splitting and enumerating one by one when solving the two-echelon spare parts stocking decision model. The authors represent the relationship between components and repair resources with a special graph, in which the vertex represents a resource and the edge represents components. The depth first search algorithm is used to find the optimal solution. The advantage of this algorithm is intuitive and easy to understand, but the disadvantage is that it needs to be enumerated one by one, and the amount of calculation is huge. Therefore, it is necessary to find a new algorithm to solve the model in this paper.

When solving the lowest spare parts stocking holding cost, a greedy heuristic algorithm is often used [28]. The authors of [10] proposed an approximate method for solving joint optimization, iterative algorithm, but they did not mention spare parts stocking decision optimization, which makes iterative algorithm difficult to solve the model in this paper. Therefore, we improve an iterative greedy heuristic algorithm [23] to solve the optimization model, as shown in Figure 3.

The article "Spare Parts Stocking Decision Strategy and Service Logistics Cost Optimization of Two-Echelon Service Logistics System considering Multifailure Mode" was retracted in 2023. Reasons: unreliable results or conclusions; concerns about the data; concerns about the peer review; concerns about the citations.

Greedy heuristic algorithm is often used in the decision-making of repairable system spare parts stocking. This algorithm can realize a fast search but can only find a local optimal solution. Iterative method is often used in joint optimization of maintenance level and spare parts allocation strategy. This algorithm traverses the whole world by iterating one by one, but it takes a long time. Combining the advantages of the above two methods, an iterative greedy heuristic algorithm is developed in this study. By iterating spare parts stocking, the local optimal solution of all spare parts allocation strategies is calculated to find the global optimal solution.

The algorithm focuses on balancing spare parts allocation and cost. According to the VAR-METRIC theory [26], we use the marginal analysis method to set the initial stocking of spare parts as 1, increase one stocking step by step until the target availability is met, and then end the algorithm. When the algorithm obtains several groups of Base and Depot stocking combinations, we select the optimal combination to guarantee the system cost.

  Step 1: set *s*_*i*,*j*_=1+*k*; *s*_*i*,0_=1+*k*.
 
*k* indicates the number of iterations. *k*=0 indicates that the initial stocking level of Base and Depot is 1.
  Step 2: set *δ*_*i*,*j*_=EBO(*s*_*i*,*j*_) − EBO(*s*_*i*,*j*_+1)/*fc*_*i*,*j*_; *δ*_*i*,0_=EBO(*s*_*i*,0_) − EBO(*s*_*i*,0_+1)/*fc*_*i*,*j*_.
 
*δ* is the marginal ability gene. It considers the marginal benefit of adding one item to the stocking [15].
  Step 3: select the best value for *δ*. Increase one unit in the stocking of item *i* at site *j*.
  Step 4: calculate the actual availability A:
 
if *A* < *A*_min_, *k* = *k* + 1, go to step 2;
 
if *A* ≥ *A*_min_, stop the calculation.
  Step 5: adjust the stocking parameter and input it into the service logistics cost optimal model.

The iterative process will produce multiple sets of spare parts stocking allocation strategy combinations, and the calculation will stop when the calculated availability is greater than the target availability, which is the local optimal solution of a combination. In this study, the local optimal solutions of all combinations are extracted, and the cost is calculated. The global optimal solution can be found from the local optimal solution.

Generally speaking, the iterative algorithm can be stopped when the availability satisfies the target availability for the first time. At this moment, the service logistics cost is the optimal cost. In order to be able to traverse the global optimal solution, iteration stops when stocking increases to the number of LRU assemblies (*M*_*i*,*j*_).

The article "Spare Parts Stocking Decision Strategy and Service Logistics Cost Optimization of Two-Echelon Service Logistics System considering Multifailure Mode" was retracted in 2023. Reasons: unreliable results or conclusions; concerns about the data; concerns about the peer review; concerns about the citations.

## 4. Numerical Experiment

### 4.1. Optimization Calculation

In this section, the energy system of a large-scale laser device is taken as an example to verify the validity of the model and algorithm. The energy system includes 96 homogeneous energy modules. Each module includes three key LRUs: Control Communication module (LRU_1_), Gas Switch module (LRU_2_), and Trigger module (LRU_3_). Due to the different tasks completed by these three LRUs, they were assigned to three different Base sites and managed by the same Depot site, as shown in Figure 4.

These three LRUs will fail randomly. In the study of large-scale system maintenance strategy, literature [29] considered the impact of failure on the delay time of system tasks when distinguishing failure mode. In this example, when distinguishing between hard failure and soft failure, we also consider the impact of failure on system task effect. We attribute the failure that leads to system task cancel to soft failure and the failure that continues to perform tasks through repair at the Base site to hard failure. The specific failure data are shown in Table 2.

Compared with soft failure, hard failure has less impact on system task results and maintenance difficulty. Therefore, the maintenance resource cost of hard failure is lower than that of soft failure. The advantage of soft failure centralized maintenance is to reduce the difficulty and cost of operating environment configuration. To ensure the execution of tasks, large-scale systems have high requirements on the availability of spare parts. We set the minimum availability requirement at 0.98. The specific parameters and cost settings of the optimization model are shown in Table 3.

Spare parts stocking decision cost, maintenance cost, and resource allocation cost of Depot are not comparable with Base. We assume that the transportation costs between the two echelons are the same, and the maintenance resources and components have a one-to-one maintenance relationship. The specific maintenance parameters are shown in Table 4.

According to the iterative greedy heuristic algorithm, we set the initial stocking allocation decision: Base (1, 1, 1) Depot (1, 1, 1). The calculated availability does not meet the requirements obviously. In the iterative process, we can get multiple sets of spare parts stocking allocation combinations. Under the constraints of limited resources, the guaranteed availability calculation results of each combination are shown in Table 5.

Extract the three groups of stocking decisions in Table 5 and calculate the service system cost by using formula (17), respectively. The results are shown in Table 6.

The article "Spare Parts Stocking Decision Strategy and Service Logistics Cost Optimization of Two-Echelon Service Logistics System considering Multifailure Mode" was retracted in 2023. Reasons: unreliable results or conclusions; concerns about the data; concerns about the peer review; concerns about the citations.

We get that the optimal cost is 214.7 ∗ 106 yuan, and the optimal stocking allocation decision is Base (3, 4, 4) Depot (1, 1, 2). The optimization result conforms to the idea of an iterative greedy heuristic algorithm. That is, when the actual availability meets the minimum requirement, the stocking allocation decision is the optimal decision. Due to the simplified optimization model, the spare parts stocking is the only variable parameter, and the optimal stocking allocation decision guarantees the optimal service logistics cost. Introducing multiple failure modes into the joint spare parts stocking decision and repair level optimization model can simplify the optimization process and make the optimization results more intuitive and easier to understand.

Combining the results in Tables 4 and 5, it can be found that when the Depot stocking level is (1, 1, 1), no matter how many times the Base stocking iterations are, it cannot satisfy the system availability requirement. This is because the stocking level of Depot plays a decisive role in the system availability. We analyze the relationship between Depot stocking level and system availability in the next section.

### 4.2. The Relationship between Depot Stocking Level between System Availability

We select the data in Table 4 and set the horizontal axis as the total stocking level S of Depot and Base. The vertical axis indicates the system availability, as shown in Figure 5.

Obviously, the improvement of stocking level is very important to improve system availability. In particular, increasing the stocking level of LRU_3_ improves the availability significantly.

Because LRU_3_ has the largest number of soft failures, it is the most difficult to repair. The optimization model will consider LRU_3_ as a key factor affecting decision-making. We can also analyze the importance of the three LRUs under different availability requirements.

### 4.3. Importance Analysis of LRUs

Under different availability requirements, the optimal stocking allocation decisions are shown in Figure 6.

It can be seen that, in the process of improving availability requirements, the ratio of LRU_3_ is always the highest. And the ratio of LRU_1_ is always the lowest. Compared with LRU_3_, LRU_1_ is the factor with the lowest EBO in Depot. Therefore, LRU_1_ has the lowest ratio in stocking allocation.

In the lower availability requirement stage (0.80∼0.93), the stocking ratio of LRU_2_ is the same as LRU_3_. In the higher availability requirement stage (0.93∼0.99), the impact of LRU_2_ on optimization decision is reduced. This means that as the difficulty of improving availability increases, the allocation of resources concentrates on the most difficult parts to repair.

The article "Spare Parts Stocking Decision Strategy and Service Logistics Cost Optimization of Two-Echelon Service Logistics System considering Multifailure Mode" was retracted in 2023. Reasons: unreliable results or conclusions; concerns about the data; concerns about the peer review; concerns about the citations.

From the above analysis, it can be seen that (1) the stocking level of the Depot plays a decisive role in ensuring the availability of the system; (2) the LRU with the highest failure rate has the highest influence on the stocking allocation decisions. In order to improve system availability, repairing time *T*_*i*,*j*_  is also a key factor that cannot be ignored.

### 4.4. Repairing Time Impact Analysis

We reduce Depot repairing time and Base repairing time, respectively. The above optimization results are reversely iterated. The changes in the availability of stocking allocation decisions are shown in Table 7.

It is obvious that reducing Depot repairing time can improve the availability of service logistics system significantly. At this point, the stocking allocation decision is Base (3, 4, 4) Depot (1, 1, 1). According to the calculation, the service logistics cost of this decision is 206.7 ∗ 106 yuan, saving 8 ∗ 106 yuan. However, the reduction of Base repairing time has little effect on the optimization results, which only shows that the availability is improved slightly. From this point of view, Depot repairing time is a key factor that could affect both system availability and service logistics cost.

Reducing Depot repairing time can save a lot of service logistics costs. However, if the Depot's maintenance capacity and stocking resources are limited, the improvement of system availability needs to consider the fronting failure mode. That is, soft failure spare parts are allocated at base site.

### 4.5. Fronting Failure Mode

Combined with Table 4 and Figure 5, we find that when the stocking level of the Depot is (1, 1, 1), no matter how to increase the stocking level of Base, the availability of the service logistics system would never meet the minimum availability requirement.

Fronting failure mode is required.

We consider the front “insulation performance degradation” of LRU_2_ and the “pilot tube performance degradation” of LRU_3_ into Base site. Their impact on the task of the operating system changes from “cancel” to “delay time.” The repairing time, spare parts stocking decision cost, and other parameters should be changed accordingly. Fronting failure mode will increase the cost of resource configuration, increase the category of spare parts at the Base maintenance point, and reassign parameters in the optimization model. The specific data are shown in Table 8.

After optimization, the stocking allocation strategy is Base (3, 3, 4) Depot (1, 1, 1), the availability is 0.9803, and the service logistics cost is 230.9 ∗ 106 yuan. Thus, if the maintenance capability of the Base could cope with soft failure mode, then the availability of the service logistics system would be improved greatly.

The article "Spare Parts Stocking Decision Strategy and Service Logistics Cost Optimization of Two-Echelon Service Logistics System considering Multifailure Mode" was retracted in 2023. Reasons: unreliable results or conclusions; concerns about the data; concerns about the peer review; concerns about the citations.

In conclusion, Depot repairing time and Base maintenance capacity are key factors affecting the service logistics system. Reducing Depot repairing time could save service logistics costs; improving Base maintenance capability could improve system availability.

## 5. Conclusion

In this paper, we construct a two-echelon service logistics cost optimization model for large-scale systems. Considering the influence of multiple failure modes on spare parts stocking decisions, the joint optimization model of spare parts stocking decision and repair level was simplified. The iterative greedy heuristic algorithm is improved to find the global optimal solution of stocking allocation strategies. Finally, the validity of the model and algorithm is verified by a practical engineering case.

The contributions and innovations of this paper are as follows: (1) Multiple failure modes are introduced into the joint optimization model to fundamentally simplify the LORA decisions and reduce the calculation process of the service logistics cost optimization. (2) The improved iterative greedy heuristic algorithm can effectively traverse the global optimal solution. (3) Depot stocking level plays a decisive role in ensuring system availability, and LRU with the highest failure rate has the highest influence on stocking allocation decisions. (4) Depot repairing time and Base maintenance capability are key factors affecting the service logistics system. Reducing Depot repairing time could save costs; improving Base maintenance capability could improve system availability.

As a further improvement, multiple failure modes would lead to discard risk. The maintenance strategy of soft failure could choose imperfect repair. A multiechelon service logistics system has a potential stocking. The increase of echelons will lead to the increase of stocking iterative combination and the complexity of the algorithm. It can be solved by an improved genetic algorithm [30, 31] and ant colony algorithm [32]. Asset management related to life cycle cost should be considered in maintenance decision-making and spare parts stocking decision management.

## Figures and Tables

**Figure 1:** The large-scale operation system with multiple failure modes.

**Figure 2:** The structure of two-echelon service logistics system.

**Figure 3:** The improved iterative greedy heuristic algorithm.

**Figure 4:** Two-echelon service logistics structure of three LRUs.

**Figure 5:** Relationship between stocking level and system availability.

The article "Spare Parts Stocking Decision Strategy and Service Logistics Cost Optimization of Two-Echelon Service Logistics System considering Multifailure Mode" was retracted in 2023. Reasons: unreliable results or conclusions; concerns about the data; concerns about the peer review; concerns about the citations.

**Figure 6:** Stocking ratio of LRUs under different availability constraints.

**Table 1:** Model variables.

*i*	Item number, LRU_*i*_, *i*=1,2,3,…, *n*
*j*	Site number, Depot: *j*=0, Base: *j*=1,2,3,…, *n*
*λ*_*i*,*j*_	Single cycle demand mean value of item *i* at site *j*
*λ*_*ih*_	Single cycle demand mean value of item *i*'s hard failure mode
*λ*_*is*_	Single cycle demand mean value of item *i*'s soft failure mode
*T*_*i*,*j*_	Repairing time of item *i* at site *j*
*O*_*i*,*j*_	Order and ship time of item *i* from the Depot to the site *j*
*fc*_*i*_	Price of item *i*
*s*_*i*,*j*_	Level of stocking of item *i* at site *j*

**Table 2:** LRUs' failure data.

Failure mode	Control communication (LRU_1_)			Gas switch (LRU_2_)			Trigger (LRU_3_)		
	Failure cause	Quantity	Influence	Failure cause	Quantity	Influence	Failure cause	Quantity	Influence
Hard failure	Communication blocking	3	Restart	Communication blocking	3	Restart	Communication blocking	1	Restart
	Software failure	3	Restart	Electromagnetic interference	3	Restart	Electromagnetic interference	1	Restart
	Electromagnetic interference	6	Restart	Barometric instability	2	Delay time	Unstable pilot tube pressure	1	Delay time

Soft failure	PLC controller damaged	3	Cancel	Insulation performance degradation	8	Cancel	Pilot tube performance degradation	10	Cancel

Total	17			16			13		

**Table 3:** LRUs' parameters.

Parameter cycle: 100 days	Depot		
	Base 1	Base 2	Base 3
	LRU_1_	LRU_2_	LRU_3_
*λ*_*i*_	17	16	13
*λ*_*ih*_	12	8	3
*λ*_*is*_	5	8	10
*T*_*i*,*j*_	0.005	0.01	0.015
*T*_*i*,0_	0.01	0.02	0.03
*O*_*i*,*j*_	0.07	0.07	0.07
*fc*_*i*,*j*_(Base)*∗*106×yuan	0.5	0.8	1
*fc*_*i*,*j*_(Depot)*∗*106×yuan	3	5	8
*M*_*i*,*j*_	96	96	192
*A*_min_	0.98		

**Table 4:** Maintenance decisions' parameters.

Maintenance decisions	Base 1	Base 2	Base 3	Depot		
	LRU_1_	LRU_2_	LRU_3_	LRU_1_	LRU_2_	LRU_3_
Repair ∗ 10^6^ yuan	1	2	3	3	5	6
Move ∗ 10^6^ yuan	1	1	1	0	0	0
*rc*_*r*,*j*_ ∗ 10^6^ yuan	3	4	5	4	6	8

**Table 5:** The system availability of different stocking allocation decisions.

Base stocking allocation	Depot stocking allocation			
	(1, 1, 1)	(1, 1, 2)	(1, 2, 2)	(1, 2, 3)
1, 1, 1	0.580867	0.614786	0.625329	0.628775
1, 1, 2	0.699793	0.73096	0.743496	0.74664
1, 2, 2	0.804553	0.840385	0.851464	0.855065
2, 2, 2	0.858257	0.896481	0.908299	0.91214
2, 2, 3	0.898131	0.933406	0.94571	0.949258
2, 3, 3	0.924175	0.960472	0.971907	0.975553
3, 3, 3	0.932103	0.968712	**0.980246**	**0.983922**
3, 3, 4	0.940104	0.975766	0.987383	0.99097
3, 4, 4	0.944344	**0.980166**	0.991567	0.995168
3, 4, 5	0.945577	0.981009	0.992419	0.996024
4, 4, 5	0.94639	0.982047	0.99347	0.997056
4, 5, 5	0.946933	0.98261	0.993996	0.997584

The article "Spare Parts Stocking Decision Strategy and Service Logistics Cost Optimization of Two-Echelon Service Logistics System considering Multifailure Mode" was retracted in 2023. Reasons: unreliable results or conclusions; concerns about the data; concerns about the peer review; concerns about the citations.

**Table 6:** The service logistics cost of different stocking allocation decisions.

Base stocking allocation			Depot stocking allocation			Service logistics cost ∗ 10^6^ yuan
**L** **R** **U**_1_	**L** **R** **U**_2_	**L** **R** **U**_3_	**L** **R** **U**_1_	**L** **R** **U**_2_	**L** **R** **U**_3_	
3	4	4	1	1	2	214.7
3	3	3	1	2	2	217.9
3	3	3	1	2	3	225.9

**Table 7:** Changes in availability for reducing repairing time.

	Base stocking allocation			Depot stocking allocation			System availability
	LRU_1_	LRU_2_	LRU_3_	LRU_1_	LRU_2_	LRU_3_	
Reduce doubled Depot repairing time	3	4	4	1	1	2	0.993372
	**3**	**4**	**4**	**1**	**1**	**1**	0.983304
	3	4	3	1	1	1	0.976317

Reduce doubled Base repairing time	3	4	4	1	1	2	0.980763
	3	3	4	1	1	2	0.977204
	3	4	3	1	1	2	0.974353

**Table 8:** Parameters after fronting failure mode.

Parameters cycle: 100 days	Base 1	Base 2	Base 3
	**L** **R** **U**_1_	**L** **R** **U**_2_	**L** **R** **U**_3_
*λ*_*i*_	17	16	13
*λ*_*ih*_	12	12	8
*λ*_*is*_	5	4	5
*T*_*i*,*j*_	0.005	0.015	0.02
*fc*_*i*,*j*_ (Base) ∗ 10^6^ yuan	0.5	1.8	2
Repair ∗ 10^6^ yuan	1	4	5
*rc*_*r*,*j*_	3	6	8

## Data Availability

The data used to support the findings of this study are included within the article.
